# Construction of the Evaluation Index System for Nurse Deployment Pertaining to the Disaster Rescue

This article has been retracted.

**DOI:** 10.1155/2022/2925689

**Published:** 2022-06-23

**Authors:** Yue Xu, Na Gao, Xiaoqian Li, Ping Wang, Haoyuan Ren, Hongying Pi

**Affiliations:** ^1^Department of Cardiology, The Second Medical Center & National Clinical Research Center for Geriatric Diseases, Chinese People's Liberation Army (PLA) General Hospital, Beijing 100853, China; ^2^The Health Service Training Center, Chinese PLA General Hospital, Beijing 100853, China

## Abstract

Based on the Delphi method, the analytic hierarchy process, and the entropy method, this paper constructs the evaluation index system for nurse deployment pertaining to the disaster rescue in military hospitals to furnish the reference evidence for scientific deployment of nursing staff, thereby promoting the rescue supportability. This paper establishes the expert consultation form of the evaluation index system for nurse deployment pertaining to the disaster rescue in military hospitals through expert interviews, group discussions, and so on. The Delphi method is applied to enquire 20 military experts in different professional fields two times, and the evaluation index system is finally determined. The weights of evaluation indexes of disaster rescue nurses are determined by the analytic hierarchy process and entropy method. The construction of the evaluation index system for the deployment of disaster relief nurses in military hospitals through Delphi method, analytic hierarchy process, and entropy method provides a reference method for rational allocation of nurses and points out the key points of hospital training. In addition, this paper provides a reference for the assessment and selection of nurses related to disaster relief in military hospitals and lays a foundation for the construction of subsequent evaluation models, which is of great significance for improving the level of nursing teams.

## 1. Introduction

The World Health Organization (WHO) believes that when any event that can cause damage to facilities, casualties, serious economic losses, threats to human health, and deterioration of social and health service conditions and the damage exceeds the extent of the area where it occurs, it cannot be tolerated. When you do not ask for help from other areas, it is a disaster [1]. Disaster events have the characteristics of complexity, destructiveness, uncertainty, and social nature and are divided into natural disasters, man-made disasters, and joint disasters [2]. They have serious adverse effects on social health, health care system, and economic development. Since the 21st century, the frequent occurrence of disasters has not only hindered the development and progress of society but also caused great loss of life and property to people all over the world.

Nurses are the largest rescue force in the front-line disaster rescue team, and they play a huge role in disaster prevention and mitigation and postdisaster rescue [3]. In the response to the Hanshin earthquake in Japan (1995), the “9.11” terrorist attack in the United States (2001), the public health emergency SARS (2003), and the Wenchuan earthquake (2008), nurses highlighted the importance of their role in disaster relief; their role has been highly appraised by the government and the public [4]. Since the outbreak of COVID-19 in 2020, more than 42,600 Chinese medical workers have been sent to Hubei to provide support and treatment, including 28,600 nurses, accounting for nearly 70% of the total, fully demonstrating that clinical nurses are increasingly becoming the main force in disaster relief. Some scholars have studied the construction of emergency disaster rescue teams and the optimal deployment of rescue teams. Arziman indicated that there is currently a lack of literature on disaster medical rescue teams, and the models of disaster medical teams in different countries in the world are different [5]. They consider the disaster medical rescue team to be a trained, mobile, self-sufficient, multidisciplinary medical team capable of providing medical services in the affected area during the acute phase of a sudden disaster, 48–72 hours after the onset of the disaster. Peller et al. conducted in-depth interviews with 10 members of the Canadian disaster medical rescue team to explore their views on the impact of nontechnical core capabilities and their own rescue experience on the speed of disaster emergency response [6]. By summarizing the experience of disaster medical rescue team members in disaster emergency management, the paper determines the nontechnical core competencies such as communication and coordination ability and cognitive ability necessary for disaster rescue response, as well as the relationship between nontechnical core competencies and professional emergency cooperation. At the same time, the importance of emergency cooperation and emergency management capabilities in the rescue process is emphasized. Leggat and Aitken [7] emphasized that government departments should ensure that members of disaster medical teams have strict selection procedures. At the same time, in terms of team training, a study on members of the Australian disaster medical team shows that more attention should be paid to the education and training of team members. At present, leadership training is considered as a necessary training content for the command and management personnel of the disaster medical team. Anan et al. [8] formulated a new training plan for disaster medical rescue teams in Japan based on Japan's earthquake relief activities and revised the training plan for disaster medical rescue teams without increasing the total training time. Evacuation, preparation of disaster medical rescue team, emergency coordination, helicopter rescue, and emergency medical information system have been added to the emergency medical rescue team training program to meet the training requirements of Japan's current disaster medical rescue team.

In China, Jiang and Li [9] believe that the selection of team members will contribute to the development of disaster medical rescue teams. In the selection of team members, not only professional skills but also personal characteristics such as personality, age, health status, experience, and teamwork should be considered.Qi [10] summarized the level of domestic disaster emergency medical rescue and the current situation of the team in recent years and improved the emergency medical rescue team by optimizing the team structure, clarifying the division of labor, strengthening professional skills training, increasing government funding, and conducting psychological intervention in a timely manner construction. Huang et al. [11], based on the experience summed up by the emergency medical rescue team in our country during the Wenchuan, Yushu, and Lushan earthquakes, believe that it is necessary to plan ahead, make adequate preparations in advance, and improve emergency response measures for various disasters, not only to strengthen emergency medical rescue. In addition to the professional training of the team, at the same time, it is necessary to do a good job in the provision of emergency rescue materials and equipment and medicines, as well as logistics support and other works. It is also necessary to strengthen the team's self-protection ability under extreme environmental conditions. Samani and Zhu [12] constantly adjusted the organizational structure of the medical personnel of the rescue team according to the occurrence law of the wounded and sick in different time periods after the earthquake, as well as the change of rescue tasks. At the same time, improving the professional and technical level of the personnel of the medical institutions in the disaster-stricken areas is proposed by taking expert guidance, unified training, and continuing education, as well as quickly restoring the functions of the medical treatment institutions in the disaster-stricken areas.

Although national experts have done a lot of research on the construction and deployment of disaster nurse teams, since the COVID-19 outbreak, countries around the world have demonstrated deficiencies in disaster preparedness. However, deployment of clinical nurses is directly related to disaster nursing ability [13–16]. Nurse deployment is the basis of rescue, and only reasonable and scientific nurse deployment can effectively treat disaster rescue and improve the quality of rescue [17–19]. Therefore, improving the deployment of clinical nurses for disaster relief and enhancing the capacity of nurses for disaster care have become the top priority at present and for quite a long time. This paper intends to establish an evaluation index system for the deployment of disaster relief nurses, in order to provide reference for the realization of scientific and reasonable deployment of nurses.

The remainder of this paper is organized as follows.  Section 2 presents the experimental method.  Section 3 provides the experimental result and Section 4 illustrates data analysis and result discussion. Finally, the conclusions of this study are given in Section 5.

## 2. The Proposed Method

### 2.1. Study Participants

The inclusion criteria of consulting experts are (1) selecting scope: military hospitals, research institute, or academies; (2) professional field: military nursing, nursing management, health service, hospital management, rescue medicine, and clinical nursing; (3) nature of work: management, research, university, and clinical; (4) professional title: the intermediate and above technical title; (5) length of employment in this field: ≥5 years, having the professional knowledge, medical theory, and practical experience, and providing comprehensive advice for this study from different perspectives; (6) willing to participate in this study; and (7) participating in the consultation constantly during the research. A total of 20 experts from Beijing, Chongqing, Shanghai, Tianjin, Sichuan, Liaoning, Shandong, and Shaanxi participated in the Delphi method-based interview. Participants are engaged in military nursing, nursing management, health service, rescue medicine, and clinical nursing. The experts in the group were 2 males and 18 females (average age: 47.25 ± 9.75 years). Most experts have senior professional titles (80%). There were 7 undergraduates, 9 M.S. degree holders, and 4 doctors. A large percentage of experts (95%) have worked for >10 years, and 40% of them had worked for >30 years.

### 2.2. Study Instruments

This paper sets up a research group, which consists of 1 head nurse, 2 assistant head nurses, and 2 head nurses. The group is mainly accountable for articulating research topics, compiling expert questionnaires, selecting consulting experts, summarizing, and analyzing the consultation results in each round. Per the research aim, we accessed literature and books and conducted field research and semistructured interviews with experts. The expert consultation questionnaire is determined after discussion in the research group. Based on the Likert five-point scoring method, each item is assigned 1–5 points from unimportant to very important. The formal expert consultation questionnaire comprised 5 first-level indicators (organization and management level, work style and quality level, technical support level, resource deployment level, and equipment support level), 23 second-level indicators, and 84 third-level indicators. Subsequently, the consultation questionnaire for the next round is finalized by the research group, and the evaluation index system of nurse deployment pertaining to the disaster rescue in military hospitals is finally established.

### 2.3. Data Collection

This paper conducts two rounds of expert consultation. The expert consultation questionnaire is distributed through mail and face to face, and it was recovered within 14 days. Afterwards, the research group analyzed the data. Following discussion, the research group decides to delete or modify the indicators whose average score of index importance is <4 or CV is >0.25. This paper selects 20 experts in related fields and invites experts to compare and score the importance of indicators at various levels in the evaluation of disaster relief nurse allocation through questionnaires and obtains a pairwise discriminant matrix.

### 2.4. Data Analysis

Quantitative data are entered into Excel and analyzed using SPSS 22.0 for Mac. This paper uses the frequency, mean, and constituent ratio for descriptive analysis and processed qualitative data using the content analysis. The following indicators reflect the expert consultation results: the recovery rate of consultation form and the proportion of experts who proposed suggestions representing the experts' enthusiasm. The MATLAB software is used to calculate the analytic hierarchy process and the entropy method, and the subjective and objective combination of weighting is used to determine the weight of each evaluation index of the disaster rescue and nursing team configuration.

## 3. The Experimental Result

### 3.1. The Delphi Expert Results of the Evaluation Index System

In two rounds, the effective recovery rate of the questionnaire is 100%, suggesting that experts supported our study and actively participated in it. Per the calculations of the Delphi method, the expert authority coefficients are 0.86. This paper applies the mean and standard deviation of importance assignment to assess the degree of concentration of experts' opinions. In the first round, the mean value of importance assignment for each index is 3.75–5.00, and the standard deviation is 0.000–0.414. In the second round, the mean value of importance assignment for each index is 4.30–4.95, and CV is 0.045–0.215, indicating that the degree of concentration of experts' opinions is high after this round and the index system formed could be adopted. The Kendall's concordance coefficients in the two rounds are 0.129 and 0.089 and demonstrated statistical significance (*P* < 0.001), suggesting that the expert opinions are well-coordinated.

### 3.2. The Consultation Results of the Evaluation Index System

#### 3.2.1. Consultation Result of the First Round

The first round comprises 5 first-level indicators, 23 second-level indicators, and 84 third-level indicators. A total of 13 experts (65%) gave suggestions, among which 6 proposed the suggestions for first-level indicators. In addition, 3 experts suggested that the “level” is not suitable for all first-level indicators and that modification is required. After discussion by the research group, the suggestion is adopted. The “I-1 organization and management level” is revised to “management efficiency”; the “I-2 team quality level” is revised to “team style and quality”; the “I-3 skill guarantee level” is revised to “professional and technical level.” One expert believed that the second- and third-level indicators under the “I-4 resource deployment level” index are primarily used to evaluate people rather than objects; after discussion, the research group adjusted them to “human resource deployment status.” Then, 3 experts believed that “I-5 equipment support level” is unsuitable for evaluating the nurse deployment pertaining to the disaster rescue in military hospitals. As nurses are not accountable for collecting and supplying equipment, this index should be deleted. One expert suggested combining “I-4 resource deployment level” and “I-5 equipment support level.” Following the discussion, “I-5 equipment support level” is deleted. For the second-level indicators, both the second-level indicators under “I-5” and the “information construction” are deleted; the latter revealed the deployment of health service units rather than the content of nursing team evaluation. The “realization function” reflected the treatment effect of the entire team and could not assess the function of the nursing team alone, which should be deleted. In addition, 1 second-level indicator “disinfection supply” is added, and 5 second-level indicators are modified (merged/transferred). For the third-level indicators, 12 indexes are added, 37 indexes are deleted, and 5 indexes are modified (merged/transferred). After the first round, the evaluation index system of nurse deployment pertaining to the disaster rescue in military hospitals is revised and formed and it included 4 first-level indicators, 20 second-level indicators, and 53 third-level indicators.

#### 3.2.2. Consultation Result of the Second Round

A total of 20 experts are invited to conduct the consultation. One expert suggested that III-10 should be added to “the scenario of desktop deduction.” “III-24 team with strong cohesion, overall view, and members who had a high sense of team identity” is revised to “members who had a high sense of team identity in department summary or job evaluation.” “III-34 average time of injury classification” is revised to “proficiency of injury classification.” Of note, these suggestions are adopted after discussion. Two experts suggested that the “qualification rate” in the third-level III-29, 30 should be changed to “qualification.”

Nevertheless, this index is designed for the entire nursing team rather than the individual nursing team; thus, this suggestion is not adopted. After two rounds of expert consultation, the evaluation index system of nurse deployment pertaining to the disaster rescue in military hospitals is finally constructed, including 4 first-level indicators, 20 second-level indicators, and 53 third-level indicators. Experts evaluated the importance of indicators at all levels, and the average score of each indicator importance is >4, and the coefficient of variation is <0.25.  Table 1 is the evaluation index system of nurse deployment pertaining to the disaster rescue in military hospitals.  Table 2 shows each index expert letter consultation score situation of nurse deployment pertaining to the disaster rescue in military hospitals.

### 3.3. Calculation of Comprehensive Weight of Evaluation Indicators for Disaster Relief Nurse Deployment

This paper uses the analytic hierarchy process and the entropy method to calculate the comprehensive weight of the evaluation index of disaster rescue nurse deployment. Through the analytic hierarchy process calculation, the indicators at all levels passed the consistency test, and the random consistency ratio (CR) is less than 0.10. The results show that the first-level indicator “professional and technical level” had the highest weight of 0.579, followed by “team style and quality” (0.178), “management efficiency” (0.141), and “manpower deployment status” (0.102). In the indicator “professional and technical level,” the secondary indicator “early treatment” has the highest weight of 0.361.  Table 3 presents the comprehensive weight of evaluation indicators for disaster relief nurse deployment.

## 4. Data Analysis and Result Discussion

Disaster rescue research in China started relatively late and is still in the exploratory stage in terms of personnel allocation and rescue capability. Due to the special mission undertaken by the army, our army has always attached great importance to the training of the disaster response capability of the medical force. However, the Wenchuan earthquake rescue operation in 2008 also exposed problems such as the low popularity of the first-aid skill training of Chinese military rescue personnel; some medical personnel are not solid enough in first aid skills. Therefore, it is emphasized to strengthen the military medical rescue capacity building and attach importance to military-local coordination. Meanwhile, it is emphasized to build nonwar military medical service through basic training and emergency medical rescue team construction.

### 4.1. Viability and Reliability of the Evaluation Index System Design

Based on the Delphi method, questionnaire survey, and expert interviews, this paper screens the indicators satisfying the evaluation of nurse deployment pertaining to the disaster rescue in military hospitals. This paper invites 20 experts to the study from different regions with regional representativeness with rich rescue support theory and practical experience, which provided a prerequisite for the reliability of the consultation results. To apply the index system to the nursing deployment pertaining to the disaster rescue in military hospitals and play an objective evaluation role, the Likert five-point rating scale is used to evaluate the index system. A CV < 0.25 suggested that expert opinions are concentrated. The statistical results illustrate that the average score of index importance in the index system is >4, and CV is <0.25, indicating that the survey objects had high recognition of the index system. Among them, the average score of index importance of four first-level indicators is >4.7. Kendall's concordance test of efficiency is statistically significant, suggestive of well-coordinated expert opinions. The results are indicative of the direction of the construction of the nursing team. The effective recovery rate of the questionnaire in two rounds is 100%, indicative of the high enthusiasm of the experts. Furthermore, the authority coefficient should be >0.7, and it is 0.86 in this study, suggesting that the authority degree is high.

### 4.2. Analysis of the Evaluation Index System of Nursing Deployment Pertaining to the Disaster Rescue in Military Hospitals

The disaster rescue and nursing security need the support of various departments and the cooperation of all nursing groups. Indeed, multiple hospitals could also be involved in the coordination and joint operations during the whole rescue procedure. Thus, standardized management will augment the cohesion of the nursing team and enhance the combat efficiency of the nursing team. Team style and quality are the key to the evaluation of the nursing team configuration. Good political quality, fine style, solid military quality, and team cooperation spirit of the nursing team depicted in daily life, training, or tasks are the prerequisite for the smooth implementation of rescue and security work. In simulated environment, training, or tasks, excellent physical and psychological qualities of nursing staff can assure the nursing work in the harsh natural climate and multifaceted environment. The professional technique affects the nursing team's rescue ability, which is the core of nursing team configuration evaluation. The nursing team's distribution and responsibilities differ in disaster rescue. The configuration includes serious injury treatment group, operation group, epidemic prevention, and elimination group. During the rescue support tasks, nursing staff in military hospitals should have the nursing responsibilities needed by the basic rules for treating the wounded. Comprehensive knowledge and excellent practical skills serve as the basis for nursing support. Human resource deployment is a direct index to reflect the evaluation of nursing team deployment. Besides, reasonable and scientific human resource deployment ability is the premise to ensure the efficiency of nursing team rescue. The number of nurses and the structure of the nursing team (e.g., personnel type, age, and professional title) are crucial components of the evaluation content of nurse deployment pertaining to the disaster rescue in military hospitals. According to the modular organization concept, the disaster rescue composition includes not only the personnel elements of the team but also the modular unit, groups, and the overall layout.

### 4.3. Calculate the Weights of Evaluation Indicators to Provide a Basis for the Subsequent Formulation of Evaluation Standards and Models for Nurse Deployment

The calculation of the index weight is very important to the process of comprehensive evaluation. This research uses the analytic hierarchy process in the subjective weighting method and the entropy value method in the objective weighting method to comprehensively calculate the weight of each index in the evaluation system. Through the analytic hierarchy process calculation, the indicators at all levels have passed the consistency test. The entropy method determines the weight under objective conditions. It can try to eliminate the subjectivity of the weighting of each factor and reflect the reliability of the indicator. However, if the difference between the indicators is large, the information entropy of the indicator will be smaller, and the weight of the indicator will be smaller. A higher value indicates the relative intensity of each index in the sense of competition, but it does not indicate the actual importance coefficient of the index. Although the analytic hierarchy process is determined based on expert scores and is subject to personal subjectivity, the determined weights of each indicator combine the profound medical practice experiences of many experts. The importance of the indicators is closer to the objective situation. Subjective and objective empowerment methods can complement each other's shortcomings and ensure the objectivity and accuracy of indicators. The research results show that the comprehensive weight of “professional and technical level (0.579)” is the highest, which has a high impact on the evaluation of the nurse deployment pertaining to the disaster rescue in military hospitals and has a more obvious impact on the evaluation of the nurse deployment; the second is the “team style and quality” (0.178), followed by “management efficiency” (0.141) and “manpower deployment status” (0.102). In the state of manpower allocation, the weight of AHP is 0.3072, which is the second largest, but, after the analysis of entropy value method, the weight of the method is the smallest, indicating that, based on expert judgment, it can be considered that manpower allocation state plays a more important role in the evaluation of nurse allocation. However, through the entropy method calculation, it is found that the differences between the three-level indicators in the manpower allocation state are small, and the effect on the evaluation of nurse allocation is small. By empowering the evaluation indicators subjectively and objectively, it provides a basis for scientifically formulating evaluation standards for the allocation of disaster relief nurses and lays a foundation for the construction of subsequent evaluation models.

## 5. Conclusion

The evaluation index system for nurse deployment pertaining to the disaster rescue in military hospitals is scientific and practical based on the Delphi method. The analytic hierarchy process and the entropy method are combined to calculate the comprehensive weight of the evaluation index to ensure the objectivity and accuracy of the index. The system provides a reference for military hospitals to reasonably allocate nurses for disaster rescue and points out the focus of the hospital training. Furthermore, this study provides a reference for the assessment and selection of nurses in military hospitals pertaining to the disaster rescue and lays a foundation for the construction of subsequent evaluation models, which is of great significance to improving the level of nursing teams.

## Figures and Tables

**Table 1:** The evaluation index system of nurse deployment pertaining to the disaster rescue in military hospitals.

First-level indicators	Second-level indicators	Third-level indicators
I-1 management efficiency	II-1 assembly principle	III-1 matching degree with rescue support mission
		III-2 matching degree with relevant standards
		III-3 matching degree with the actual hospital condition
	II-2 planning organization	III-4 completing the nursing plan within a specified time
		III-5 complete and accurate nursing elements in the program with solid pertinence and operability
		III-6 modifying and revising the plan according to the changing tasks
	II-3 controlling coordination	III-7 complete and well-implemented nursing system during the task implementation
		III-8 the nursing force could be adjusted reasonably and well cooperated
		III-9 cooperating with relevant departments actively
	II-4 auxiliary decision-making	III-10 strong information processing capability and practical judgment of the nursing information in the desktop deduction and other scenarios
		III-11 nursing managers with more than 5 years of practical rescue experience and nursing professional guidance capability
		III-12 strong capability to deal with emergencies and reasonable and feasible nursing suggestions
	II-5 organizational training	III-13 independent or comprehensive nursing annual plan and exercise program in line with the relevant provision
		III-14 nursing staff training, rehearsed plan with the detailed record for further evaluation and summary

I-2 team style and quality	II-6 ideological style	III-15 firm political stance, a strong sense of responsibility and mission, and no disciplinary action
		III-16 the revolutionary spirit of selfless dedication and fine style, the experience of participating in the implementation of urgent, difficult, dangerous, and heavy tasks or commendation in daily work
		III-17 the sense of patient care, good self-cultivation, and high service satisfaction in daily security
	II-7 military physical fitness	III-18 qualification rate of military theory assessment
		III-19 qualification rate of military physical fitness assessment based on the assessment standard of “training program”
		III-20 qualification rate of rescue training personnel in recent three years
	II-8 environmental adaptation	III-21 excellent psychological quality and acclimatization training in a particular environment
		III-22 participating in continuous operation training or task under high intensity or complex environment
		III-23 mastering the survival skills in the field
	II-9 teamwork	III-24 members with a high sense of team identity in the department summary or job evaluation
		III-25 smooth communication and good cooperation between the internal and external during the training
	II-10 emergency response	III-26 definite plan of nursing staff collection and timely and orderly assembly
		III-27 rapid and orderly nursing staff who are responsible for loading and unloading goods and materials
		III-28 quick and orderly nursing staff during the withdrawal

I-3 professional and technical level	II-11 early treatment	III-29 qualification rate of nursing theory examination on early treatment items stipulated in the wounded treatment rules
		III-30 qualification rate of nursing operation skill examination in the main items of early treatment
		III-31 proportion of nursing staff who could complete the general debridement independently
	II-12 specific treatment	III-32 qualification rate of nursing theory examination on specialized treatment items stipulated in the wounded treatment rules
		III-33 qualification rate of nursing operation skill examination on significant items of specialized treatment
	II-13 classification during the evacuation	III-34 proficiency in injury classification
		III-35 accuracy rate of nursing operation in injury classification
		III-36 qualification rate of nursing skill examination on emergency treatment of injuries during the evacuation
	II-14 disinfection supply	III-37 qualification rate of theoretical examination on ishing, disinfection, and sterilization
		III-38 qualification rate of technical examination on disinfection and sterilization of instruments and objects
	II-15 epidemic prevention and protection	III-39 qualification rate of theoretical examination on the epidemic prevention and health protection
		III-40 qualification rate of technical examination on the diet, drinking, isolation, and environmental disinfection skills of the wounded
		III-41 qualification rate of technical examination on detection and decontamination of nuclear chemical wounded
	II-16 the usage of medical equipment	III-42 the operation process specification and proficiency of nursing equipment
		III-43 basic maintenance skills of nursing equipment
	II-17 medical information processing	III-44 timely and accurate medical information collection report
		III-45 skilled use of postinformation medical equipment

I-4 manpower deployment status	II-18 deployment status	III-46 reasonable deployment of the number of nursing staff in the rescue team
		III-47 the coordination degree between the number of rescue nurses in the rescue team and the nursing establishment of the hospital
	II-19 deployment structure	III-48 meeting the requirements of the military configuration ratio
		III-49 meeting the requirements of the medical staff configuration ratio
		III-50 meeting the requirements of middle and senior nursing technical staff configuration ratio
		III-51 meeting the requirements of the age structure deployment ratio
	II-20 personnel distribution	III-52 reasonable degree of nursing staff deployment
		III-53 reasonable degree of nursing unit module organization

**Table 2:** Each index expert letter consultation score situation of nurse deployment pertaining to the disaster rescue in military hospitals.

Indicators	Degree of importance					Mean	Standard deviation	Coefficient of variance
	5 points	4 points	3 points	2 points	1 point			
I-1 management efficiency	15 (75)	4 (20)	1 (5)	—	—	4.70	0.571	0.121
II-1 assembly principle	16 (80)	3 (15)	1 (5)	—	—	4.80	0.410	0.085
III-1	18 (90)	1 (5)	1 (5)	—	—	4.85	0.489	0.101
III-2	15 (75)	4 (20)	1 (5)	—	—	4.75	0.444	0.093
III-3	13 (65)	4 (20)	3 (15)	—	—	4.75	0.550	0.116
II-2 planning organization	19 (95)	—	1 (5)	—	—	4.90	0.447	0.091
III-4	17 (85)	1 (5)	2 (10)	—	—	4.70	0.733	0.156
III-5	17 (85)	2 (10)	1 (5)	—	—	4.65	0.489	0.105
III-6	17 (85)	1 (5)	2 (10)	—	—	4.75	0.910	0.192
II-3 controlling coordination	16 (80)	3 (15)	—	1 (5)	—	4.65	0.671	0.144
III-7	16 (80)	3 (15)	1 (5)	—	—	4.75	0.444	0.093
III-8	15 (75)	4 (20)	1 (5)	—	—	4.85	0.366	0.075
III-9	15 (75)	4 (20)	1 (5)	—	—	4.85	0.366	0.075
II-4 auxiliary decision-making	13 (65)	7 (35)	—	—	—	4.90	0.308	0.063
III-10	15 (75)	4 (20)	1 (5)	—	—	4.95	0.224	0.045
III-11	12 (60)	5 (25)	3 (15)	—	—	4.95	0.224	0.045
III-12	15 (75)	5 (25)	—	—	—	4.80	0.523	0.109
II-5 organizational training	18 (90)	1 (5)	—	—	1 (5)	4.80	0.410	0.085
III-13	14 (70)	5 (25)	1 (5)	—	—	4.80	0.410	0.085
III-14	16 (80)	3 (15)	1 (5)	—	—	4.85	0.366	0.075
I-2 team style and quality	16 (80)	4 (20)	—	—	—	4.75	0.444	0.093
II-6 ideological style	15 (75)	3 (15)	2 (10)	—	—	4.80	0.523	0.109
III-15	18 (90)	2 (10)	—	—	—	4.65	0.813	0.175
III-16	17 (85)	3 (15)	—	—	—	4.70	0.571	0.121
III-17	17 (85)	3 (15)	—	—	—	4.85	0.489	0.101
II-7 military physical fitness	15 (75)	5 (25)	—	—	—	4.70	0.571	0.121
III-18	15 (75)	4 (20)	1 (5)	—	—	4.50	0.761	0.169
III-19	17 (85)	2 (10)	1 (5)	—	—	4.75	0.639	0.135
III-20	12 (60)	7 (35)	1 (5)	—	—	4.80	0.523	0.109
II-8 environmental adaptation	17 (85)	3 (15)	—	—	—	4.75	0.639	0.135
III-21	16 (80)	4 (20)	—	—	—	4.75	0.550	0.116
III-22	12 (60)	7 (35)	1 (5)	—	—	4.70	0.571	0.121
III-23	14 (70)	5 (25)	1 (5)	—	—	4.70	0.571	0.121
II-9 teamwork	17 (85)	3 (15)	—	—	—	4.70	0.571	0.121
III-24	18 (90)	2 (10)	—	—	—	4.45	0.759	0.171
III-25	18 (90)	2 (10)	—	—	—	4.75	0.444	0.093
II-10 emergency response	18 (90)	2 (10)	—	—	—	4.65	0.587	0.126
III-26	16 (80)	3 (15)	1 (5)	—	—	4.75	0.550	0.116
III-27	15 (75)	3 (15)	2 (10)	—	—	4.90	0.308	0.063
III-28	15 (75)	4 (20)	1 (5)	—	—	4.85	0.366	0.075
I-3 professional and technical level	18 (90)	1 (5)	1 (5)	—	—	4.85	0.366	0.075
II-11 early treatment	19 (95)	1 (5)	—	—	—	4.70	0.571	0.121
III-29	13 (65)	5 (25)	2 (10)	—	—	4.80	0.523	0.109
III-30	15 (75)	3 (15)	2 (10)	—	—	4.55	0.605	0.133
III-31	13 (65)	6 (30)	1 (5)	—	—	4.80	0.410	0.085
II-12 specific treatment	19 (95)	1 (5)	—	—	—	4.55	0.605	0.133
III-32	13 (65)	6 (30)	1 (5)	—	—	4.65	0.587	0.126
III-33	15 (75)	4 (20)	1 (5)	—	—	4.90	0.308	0.063
II-13 classification during the evacuation	18 (90)	1 (5)	1 (5)	—	—	4.90	0.308	0.063
III-34	15 (75)	5 (25)	—	—	—	4.75	0.550	0.116
III-35	18 (90)	1 (5)	1 (5)	—	—	4.65	0.671	0.144
III-36	16 (80)	4 (20)	—	—	—	4.70	0.571	0.121
II-14 disinfection supply	16 (80)	4 (20)	—	—	—	4.55	0.686	0.151
III-37	13 (65)	6 (30)	1 (5)	—	—	4.65	0.671	0.144
III-38	15 (75)	4 (20)	—	1 (5)	—	4.60	0.598	0.130
II-15 epidemic prevention and protection	16 (80)	4 (20)	—	—	—	4.60	0.598	0.130
III-39	12 (60)	8 (40)	—	—	—	4.70	0.571	0.121
III-40	15 (75)	5 (25)	—	—	—	4.75	0.444	0.093
III-41	14 (70)	4 (20)	2 (10)	—	—	4.85	0.489	0.101
II-16 the usage of medical equipment	17 (85)	3 (15)	—	—	—	4.80	0.410	0.085
III-42	17 (85)	2 (10)	1 (5)	—	—	4.60	0.598	0.130
III-43	13 (65)	5 (25)	2 (10)	—	—	4.65	0.745	0.160
II-17 medical information processing	15 (75)	5 (25)	—	—	—	4.60	0.503	0.109
III-44	15 (75)	5 (25)	—	—	—	4.75	0.444	0.093
III-45	15 (75)	5 (25)	—	—	—	4.60	0.681	0.148
I-4 manpower deployment status	15 (75)	5 (25)	—	—	—	4.80	0.523	0.109
II-18 deployment status	17 (85)	2 (10)	1 (5)	—	—	4.55	0.686	0.151
III-46	15 (75)	5 (25)	—	—	—	4.75	0.444	0.093
III-47	12 (60)	7 (35)	1 (5)	—	—	4.75	0.444	0.093
II-19 deployment structure	16 (80)	2 (10)	1 (5)	1 (5)	—	4.75	0.444	0.093
III-48	11 (55)	5 (25)	3 (15)	1 (5)	—	4.55	0.605	0.133
III-49	16 (80)	4 (20)	—	—	—	4.30	0.923	0.215
III-50	11 (55)	7 (35)	2 (10)	—	—	4.80	0.410	0.085
III-51	14 (70)	4 (20)	2 (10)	—	—	4.45	0.686	0.154
II-20 personnel distribution	15 (75)	4 (20)	1 (5)	—	—	4.60	0.681	0.148
III-52	14 (70)	5 (25)	1 (5)	—	—	4.65	0.587	0.126
III-53	14 (70)	4 (20)	1 (5)	1 (5)	—	4.55	0.826	0.182

**Table 3:** Comprehensive weight of evaluation indicators for disaster relief nurse deployment.

Indicators	Analytic hierarchy process weight	Entropy method weight	The comprehensive weights
I-1 management efficiency	0.1479	0.247821	0.141
II-1 assembly principle	0.0793	0.191427	0.077
III-1	0.3338	0.567643	0.575
III-2	0.41	0.190929	0.237
III-3	0.2562	0.241428	0.188
II-2 planning organization	0.2073	0.187759	0.199
III-4	0.1802	0.302807	0.171
III-5	0.3495	0.519874	0.568
III-6	0.4703	0.17732	0.261
II-3 controlling coordination	0.2235	0.240516	0.274
III-7	0.2124	0.372947	0.231
III-8	0.4671	0.427476	0.582
III-9	0.3205	0.199577	0.187
II-4 auxiliary decision-making	0.1696	0.223047	0.193
III-10	0.1324	0.292362	0.118
III-11	0.2087	0.392942	0.250
III-12	0.6589	0.314696	0.632
II-5 organizational training	0.3203	0.157251	0.257
III-13	0.3214	0.499985	0.321
III-14	0.6786	0.500015	0.679
I-2 team style and quality	0.1849	0.249126	0.178
II-6 ideological style	0.0883	0.113959	0.055
III-15	0.2629	0.272498	0.195
III-16	0.5674	0.43128	0.667
III-17	0.1697	0.296222	0.137
II-7 military physical fitness	0.1222	0.243718	0.163
III-18	0.1808	0.333514	0.181
III-19	0.4022	0.322489	0.389
III-20	0.4171	0.343997	0.430
II-8 environmental adaptation	0.145	0.306745	0.243
III-21	0.2591	0.466277	0.351
III-22	0.3191	0.01241	0.011
III-23	0.4218	0.521313	0.638
II-9 teamwork	0.2391	0.224085	0.293
III-24	0.4891	0.50104	0.490
III-25	0.5109	0.49896	0.510
II-10 emergency response	0.4053	0.111494	0.247
III-26	0.2714	0.372348	0.302
III-27	0.2551	0.290574	0.221
III-28	0.4736	0.337078	0.477
I-3 professional and technical level	0.36	0.417024	0.579
II-11 early treatment	0.2645	0.198212	0.361
III-29	0.2109	0.333456	0.211
III-30	0.3958	0.357757	0.425
III-31	0.3933	0.308787	0.364
II-12 specific treatment	0.1169	0.193927	0.156
III-32	0.3435	0.5000	0.344
III-33	0.6565	0.5000	0.657
II-13 classification during the evacuation	0.193	0.071333	0.095
III-34	0.2995	0.177307	0.159
III-35	0.3881	0.306734	0.357
III-36	0.3123	0.515959	0.483
II-14 disinfection supply	0.0942	0.171916	0.112
III-37	0.3782	0.500035	0.378
III-38	0.6218	0.499965	0.622
II-15 epidemic prevention and protection	0.1233	0.186167	0.158
III-39	0.219	0.311034	0.207
III-40	0.4448	0.268941	0.364
III-41	0.3362	0.420025	0.429
II-16 The usage of medical equipment	0.1231	0.053683	0.046
III-42	0.6527	0.500053	0.653
III-43	0.3473	0.499947	0.347
II-17 medical information processing	0.085	0.124762	0.073
III-44	0.5056	0.499913	0.506
III-45	0.4944	0.500087	0.494
I-4 manpower deployment status	0.3072	0.086029	0.102
II-18 deployment status	0.2512	0.349592	0.262
III-46	0.6929	0.500017	0.693
III-47	0.3071	0.499983	0.307
II-19 deployment structure	0.3944	0.417171	0.491
III-48	0.0776	0.247851	0.081
III-49	0.2436	0.372392	0.381
III-50	0.3157	0.211328	0.281
III-51	0.3631	0.168429	0.257
II-20 personnel distribution	0.3545	0.233238	0.247
III-52	0.3982	0.499951	0.398
III-53	0.6018	0.500049	0.602

## Data Availability

The simulation experiment data used to support the findings of this study are available from the corresponding author upon request.
